The article "Repetitive Transcranial Magnetic Stimulation Improves Neuropathy and Oxidative Stress Levels in Rats with Experimental Cerebral Infarction through the Nrf2 Signaling Pathway" was retracted in 2023. Reasons: signs of a paper mill; compromised peer review; unreliable results or conclusions.

# Repetitive Transcranial Magnetic Stimulation Improves Neuropathy and Oxidative Stress Levels in Rats with Experimental Cerebral Infarction through the Nrf2 Signaling Pathway

**DOI:** 10.1155/2021/3908677

**Published:** 2021-09-06

**Authors:** Hui Liang, Congjie Xu, Shijun Hu, Gang Wen, Jie Lin, Tao Liu, Jiyi Xu

**Affiliations:** ^**1**^ Department of Neurology, Hainan General Hospital, Hainan Affiliated Hospital of Hainan Medical University, Haikou, Hainan 570311, China; ^**2**^ Department of Urology, Hainan General Hospital, Hainan Affiliated Hospital of Hainan Medical University, Haikou, Hainan 570311, China; ^**3**^ Department of Emergency, Nanfang Hospital, Southern Medical University, Guangzhou, Guangdong 510515, China; ^**4**^ The National Clinical Research Center for Mental Disorders & Beijing Key Laboratory of Mental Disorders, Beijing Anding Hospital, Capital Medical University, Beijing 100088, China; ^**5**^ Advanced Innovation Center for Human Brain Protection, Capital Medical University, Beijing 100088, China

## Abstract

Ischemic stroke poses a serious threat to human health. Its high morbidity, disability, and lethality rates have led to it being a research hotspot. Cerebral ischemia reperfusion injury is a difficult point in the treatment of ischemic stroke. In recent years, studies have shown that repeated transcranial magnetic stimulation (rTMS) can enhance cerebral ischemic tolerance and have a significant protective effect on reperfusion injury after ischemia, but its specific mechanism is unknown. The Nrf2/pathway plays a vital role in ischemia-reperfusion injury in the body environment. Therefore, in this experiment, the middle cerebral artery occlusion (MCAO) reperfusion model of SD rats was made to simulate the occurrence of experimental cerebral infarction by the suture method. After treatment with rTMS, it was studied whether it can regulate the expression of Nrf2 and HO-1, affect the content of MDA and SOD activity, and then activate the Nrf2 pathway to exert its brain protection. The results showed that after MCAO reperfusion, the neurological deficit score of rats increased, and the time to remove the bilateral stickers and the time to cross the balance beam increased, suggesting the successful establishment of the experimental cerebral infarction model. Detecting the brain tissue of experimental cerebral infarction rats found that the expression of Nrf2 and HO-1 decreased, the content of MDA increased, and the activity of SOD decreased. After rTMS treatment, the neuromotor function of experimental cerebral infarction rats improved, the expression of Nrf2 and HO-1 in the brain tissue gradually increased, the content of MDA decreased, and the activity of SOD increased. It indicates that the expression of Nrf2 and HO-1 in experimental cerebral infarction rats is reduced. After treatment with rTMS, it can improve the neuromotor function damage of the rats and reduce the level of oxidative stress. The mechanism may be through promoting the activation of the Nrf2 signaling pathway, acting on the expression of antioxidant proteins, such as HO-1 and SOD1, reducing oxidative stress damage, and playing a protective effect on brain tissue.

## 1. Introduction

Cerebral infarction, also known as ischemic stroke, is due to the interruption of blood supply to the brain, resulting in the lack of oxygen and glucose supply in the brain tissue, resulting in focal tissue necrosis and softening. It is characterized by high incidence and high fatalities, disability rate, high recurrence rate, and high fatality rate, and it is becoming younger and younger [1]. At present, for the treatment of ischemic stroke, we prefer thrombolytic therapy in the acute treatment time window. However, thrombolytic therapy produces a series of side effects while recanalizing the blood vessels. The most difficult one is cerebral ischemia-reperfusion injury [2]. The core pathological links of ischemia-reperfusion injury mainly include oxidative stress damage and the chain reaction of free radicals [3]. Therefore, the main methods for the treatment of ischemic encephalopathy include antioxidative stress therapy, blocking the cascade of cerebral ischemic damage and reducing neuronal damage in the ischemic penumbra. Oxidative stress is a pathological process in which the body produces excessive reactive oxygen free radicals (ROS) when subjected to various harmful stimuli to cause endogenous antioxidant reactions. This imbalance leads to the accumulation of oxidative damage, including modification of lipids, proteins, and nucleic acids after translation. The brain is particularly vulnerable to oxidative damage due to its high lipid content and high oxygen consumption. During cerebral ischemia-reperfusion injury, a large amount of ROS products will be produced. The large increase in ROS products will aggravate ischemia-reperfusion injury in many ways, including blood-brain barrier destruction, inflammation, and apoptosis. Interfering with the mitochondrial respiratory chain will produce a large amount of superoxide anion free radicals [4]. Inhibiting the generation of ROS through genes or pharmacological mechanisms can protect the brain tissue after stroke, reduce the destruction of the blood-brain barrier, and reduce inflammation [5]. Malondialdehyde (MDA) is a metabolite of the body's peroxidation reaction triggered by oxygen free radicals, which can reflect the degree of cell damage. As a natural antioxidant enzyme, superoxide dismutase (SOD) can scavenge ROS in the body, and its activity reflects the body's ability to scavenge oxygen free radicals [6].

Nuclear transcription factor E2-related factor 2 (Nrf2) belongs to the Cap-n-collar (CNC) leucine zipper transcription factor family. It consists of 589 amino acids and contains 6 highly conserved domains Neh (Neh1–Neh6) [7]. Under physiological conditions, Nrf2 and Keap1 bind stably in the cytoplasm and are in an inactive state. When oxidative stress occurs, Nrf2 dissociates from Keap1, and Nrf2 enters the nucleus to combine with antioxidant response elements (ARE) [8], activate downstream related genes, and promote the expression of a variety of enzymes and nonenzyme antioxidant genes, including heme oxygenase 1 (HO-1), SOD, glutathione peroxidase, quinone oxidoreductase 1 (NQO-1), and catalase (CAT), to enhance cell resistance to oxidative damage stress ability [9]. Some studies [10] believe that the use of Nrf2, an excitatory drug, pinacidil, can significantly increase the antioxidative stress of the cardiology and improve myocardial function. The mechanism is that the expression of Nrf2 protein is upregulated after the above treatment, thereby activating the Nrf2/ARE pathway, exerting its antioxidative stress effect. Another study [11] showed that the use of the electrophile NEPP as the activator of the Nrf2/ARE pathway to activate the Nrf2/ARE pathway can upregulate a variety of downstream antioxidant enzymes in the cerebral ischemia reperfusion model, confirming that the Nrf2/ARE pathway has a protective effect on the brain.

Repetitive transcranial magnetic stimulation (rTMS) is a new neuroelectrophysiological technology developed on the basis of transcranial magnetic stimulation in 1992. It can affect the function of local and distant cortex, realize functional regional reconstruction, and affect the expression of a variety of neurotransmitters and gene levels [12]. At present, it has gradually been used in treatment research, and it has been proved to have a definite effect on neuropsychiatric diseases such as major depression and movement disorders [13]. In recent years, rTMS has been gradually used in more and more studies to treat ischemic cerebrovascular disease, confirming that rTMS can promote the recovery of exercise, learning, and memory in patients with cerebral infarction and promote the reduction of neurological function scores in rats with cerebral ischemia reperfusion [14]. It has an obvious protective effect on brain injury after ischemia and reperfusion, but its specific mechanism is unknown. This experiment will establish a transient occlusion (middle cerebral artery occlusion, MCAO) model of the right middle cerebral artery and observe the effect of rTMS on neuromotor function changes in MCAO rats. Analyze the expression of Nrf2 and HO-1 in the ischemic brain tissue and the influence of MDA content and SOD activity in the ischemic brain tissue homogenate to explore whether rTMS can activate the Nrf2/ARE signal pathway to achieve neuroprotection. The specific report is as follows.

## 2. Materials and Methods

### 2.1. Animal Grouping and Animal Model Preparation

Forty-five adult male SD rats (250 g–280 g) (Jiangsu Ailingfei Biological Technology Co., Ltd.) were randomly assigned to 3 experimental groups according to the principle of random allocation, namely, the sham group, the model group, and the rTMS treatment group, with 15 rats in each group. The MCAO reperfusion model was made by the suture method. The sham group used the same operation but did not insert the suture. The rTMS treatment group began to intervene with rTMS on the first day after surgery, until 14 days after surgery, stimulate at the same time point every day, stimulate 3 groups every day, each group has 20 sequences, each sequence is separated by 1 s, and each group is separated by 1 minute. In the model group, sham rTMS was used to stimulate the MCAO model [15] SD rats under the same conditions.

### 2.2. Specific Tests

#### 2.2.1. Neurological Function Score

Refer to Longa's 5-point system [16] to evaluate neurological function after 24 hours of ischemia-reperfusion: 0 points, no symptoms of neurological injury; 1 point, mild focal neurological deficit (the paralyzed anterior and hind limbs cannot be fully extended); 2 points, moderate focal neurological deficit (circle to the paralyzed side); 3 points, severe neurological deficit (dumping to the paralyzed side while crawling); 4 points, unable to go spontaneously, loss of consciousness; and 5 points, cannot walk at all. Based on the points in the above situation, the cumulative score will be the final score.

#### 2.2.2. Motor Function Evaluation

The motor function was evaluated by the double-sided sticker removal experiment and the balance beam walking experiment. Double-sided sticker removal experiment: 14 days after the animal operation, two pieces of square adhesive paper with a side length of 10 mm were used to stick the palm surfaces of the two forelimbs of the rat (the degree of viscosity is preferably when the adhesive paper is bitten off within 10 s of a normal rat), and the rat was placed in the test cylinder. The rat will instinctively bite off the paper. Observe and record the total time for the rat to remove the paper on both sides. If the paper is not removed within 120 s, it is recorded as 120 s. Balance beam walking experiment: the experiment was carried out 14 days after the operation. The balance beam was 105 cm × 4 cm × 3 cm wooden strips. Both ends were fixed, so that the wooden strips were 80 cm off the ground. The starting point was a steep platform, and the end point was a platform to record the time that the rats' limbs passed the entire balance beam. Failure to pass the entire balance bar for more than 120 s is recorded as 120 s, and a rat falling from the balance bar is recorded as a failure for more than 120 s. Before the test, the rats are trained once a day for a total of 2 days.

#### 2.2.3. Preparation of Tissue Specimens

After the rats in each group were anesthetized, the thoracic cavity was opened under the xiphoid process, and the aortic arch was intubated from the apex of the heart, and the right atrial appendage was cut open. Approximately 500 mL of sterile normal saline was used for perfusion and flushing until the color was clear, and 500 mL of 4% paraformaldehyde was used for perfusion until the whole body was stiff. Then, the brain was taken and placed in 4% paraformaldehyde solution and fixed at 4°C for 24 h. After embedding in conventional dehydrated paraffin blocks, a tissue slicer (Leica, Germany) was used to make serial coronal slices at the bregma position (the site of cerebral infarction) with a thickness of 2–5 *μ*m. The brain slices were stored in a refrigerator at −20°C.

#### 2.2.4. Western Blot Protein Quantification

The total protein of rat brain tissue was extracted, and the total protein concentration was determined with the BCA protein concentration determination kit. After electrophoresis, membrane transfer, blocking, and the addition of corresponding antibodies Nrf2 (1 : 1000), HO-1 (1 : 1000), and *β*-actin (1 : 1000), the expression levels of Nrf2 and HO-1 protein in each group were detected.

#### 2.2.5. RT-PCR

The expression of Nrf2 and HO-1 was determined by the RT-PCR method. The total RNA was extracted with TRIzol reagent, the amount of RNA was measured by UV spectrophotometer, and the RNA was reverse transcribed into cDNA, and then, PCR reaction was performed to perform PCR amplification of the corresponding target genes. The specific primer sequences are given in Table 1. 2^−ΔΔCt^ was used to calculate the relative mRNA expression of the target gene.

#### 2.2.6. Detection of SOD Activity and MDA Content in Brain Tissue

Strictly follow the instructions of the ELISA kit. The absorbance value was measured at 450 nm wavelength with an enzyme-linked instrument, and the mass concentration of SOD and MDA in the sample was calculated by drawing a standard curve.

### 2.3. Statistical Analysis

SPSS17.0 software was used for statistical analysis. The result was expressed as ($\bar{x}\pm s$). For measurement data, analysis of variance was used, and for count data, the chi-square test was used. Test level *α* = 0.05, two-sided test, *p* < 0.05 indicates statistical difference.

## 3. Results

### 3.1. The Effect of Cerebral Ischemia-Reperfusion on Neuromotor Injury in Rats

The neuromotor function evaluation results showed that compared with the sham group, the neurological deficit score of the model group increased, and the time for removing the bilateral stickers and the time for the balance beam are to be increased. The differences were statistically significant (*p* < 0.05). It suggests that the experimental rat model of cerebral infarction has been successfully established, as shown in Figures 1(a) and 1(b).

### 3.2. The Expression of Nrf2 and HO-1 and the Level of Oxidative Stress in the Brain Tissue of Experimental Cerebral Infarction Rats

Western blot and RT-PCR detection of the expression of Nrf2 and HO-1 in the brain tissue of experimental cerebral infarction rats found that compared with the sham group, the expression of Nrf2, HO-1 protein, and mRNA in the brain tissue of the model group was reduced. The differences were statistically significant (*p* < 0.05), as shown in Figures 2(a)–2(d). The oxidative stress test found that the SOD level in the brain tissue of the model group decreased and the MDA level increased. The differences were statistically significant (*p* < 0.05), as shown in Figures 2(e) and 2(f).

### 3.3. The Effect of Repeated Transcranial Magnetic Stimulation on the Neuromotor Function of Rats with Experimental Cerebral Infarction

The neuromotor function evaluation results showed that compared with the model group, the neurological deficit score of the rTMS treatment group was reduced, and the time for removing the bilateral stickers and the time for balance beam passing time were reduced. The differences were statistically significant (*p* < 0.05). It is suggested that rTMS can improve the neuromotor function of rats with experimental cerebral infarction, as shown in Figures 3(a) and 3(b).

### 3.4. The Effect of Repeated Transcranial Magnetic Stimulation on the Expression of Nrf2 and HO-1 in the Brain Tissue of Experimental Cerebral Infarction Rats

Western blot and RT-PCR detection of the expression of Nrf2 and HO-1 in the brain tissue of experimental cerebral infarction rats found that compared with the model group, the expression of Nrf2, HO-1 protein, and mRNA in the brain tissue of the rTMS treatment group increased. The differences were statistically significant (*p* < 0.05), as shown in Figures 4(a)–4(d).

### 3.5. The Effect of Repeated Transcranial Magnetic Stimulation on Oxidative Stress in the Brain Tissue of Experimental Cerebral Infarction Rats

The oxidative stress test found that compared with the model group, the SOD level in the brain tissue of the rTMS treatment group increased and the MDA level decreased. The differences were statistically significant (*p* < 0.05), as shown in Figures 5(a) and 5(b).

## 4. Discussion

Cerebral infarction refers to ischemic necrosis or softening of brain tissue, leading to cerebral blood circulation disorders and tissue ischemia and hypoxia. The prognosis is good for mild cases and life-threatening in severe cases. Cerebral infarction is the most common type of cerebrovascular diseases, accounting for about 70% of all acute cerebrovascular diseases, and it is more common in middle-aged and elderly patients [17]. According to recent studies, the disease is getting younger and younger and has a serious impact on the development of society [18]. In the treatment of cerebral infarction, cerebral ischemia reperfusion injury is often caused. The mechanism of cerebral ischemia-reperfusion injury includes excitatory amino acid toxicity, massive generation of oxygen free radicals, intracellular calcium ion overload, mitochondrial damage, cell apoptosis, and immune inflammatory damage [19–21]. Oxygen free radicals are one of the mechanisms that cause ischemia-reperfusion injury. In neurodegenerative diseases, iron accumulation in mitochondria leads to oxidative stress damage. In recent years, oxidative stress has received widespread attention as the main link of cerebral ischemia and reperfusion.

The Nrf2 pathway is the most important antioxidative stress system in the body [22]. HO-1 is an important heme-degrading enzyme with anti-inflammatory and antiapoptotic effects [23]. In our study, it was found that after MCAO reperfusion, the neurological deficit score of rats increased, and the time for removing the bilateral stickers and the time for the balance beam to cross the rod increased, suggesting that the rat neuromotor function is abnormal, and the experimental cerebral infarction rat model was successfully established. Detecting the expression of Nrf2 and HO-1 in the brain tissue of experimental cerebral infarction rats found that the expression of Nrf2, HO-1 protein, and mRNA in the brain tissue of the model group decreased, indicating that in the brain tissue of experimental cerebral infarction rats, Nrf2, HO-1 is at a low level. HO-1 is a stress protein related to the iron metabolism. HO-1 can decompose heme into biliverdin CO and iron. Under stress, it can protect against oxidative stress. However, when it is chronically overexpressed, it can promote iron deposition and generate more toxic hydroxyl radicals through the Fenton reaction [24]. Oxidative stress detection found that the SOD level in the brain tissue of experimental cerebral infarction rats decreased, and the MDA level increased, indicating that there is a serious oxidative stress phenomenon in the brain tissue of experimental cerebral infarction rats. Cerebral ischemia and reperfusion injury can cause a large amount of ROS in the body. The speed and activity of SOD catalase and other antioxidant enzymes to neutralize ROS are limited, causing ROS imbalance; unreduced ROS will cause serious oxidative damage to cell membranes. MDA is one of the end products of this process [25].

rTMS has been found to promote the recovery of exercise, learning, and memory in patients with cerebral infarction and to improve neurological damage in rats with cerebral ischemia and reperfusion [26, 27]. In our experiments, it was found that in rats treated with rTMS, the neurological deficit scores were reduced, and the time to remove bilateral stickers and the time to cross the balance beam was reduced, which confirmed that rTMS can improve the neuromotor function of rats with experimental cerebral infarction. Through observation, we also found that the expression of Nrf2, HO-1 protein, and mRNA in the brain tissue of rats in the rTMS treatment group increased, the level of SOD increased, and the level of MDA decreased. It is suggested that rTMS can induce the activation of the Nrf2 pathway, increase the level of HO-1, and improve the oxidative stress response. This may be because both ischemic injury and ischemia-reperfusion injury can cause the body's oxidative stress response, and the Nrf2 pathway serves as a defensive signal transduction pathway for the body to resist internal and external oxidation and stimulation. The endogenous antioxidant response mechanism plays a role in the process of oxidative stress [28]. When the body responds to oxidative stress, Nrf2 can be rapidly phosphorylated and activated and transferred to the nucleus. By acting on the downstream ARE protein, it can promote the expression of antioxidant proteins such as HO-1 and SOD1, inhibit the expression of MDA, and relieve the brain tissue. Oxidative stress damage is caused by excessive ROS [29].

## 5. Conclusion

The expression of Nrf2 and HO-1 decreased in experimental cerebral infarction rats. After treatment with rTMS, it can improve the neuromotor function damage and reduce the level of oxidative stress in rats. The mechanism may be through promoting the activation of the Nrf2 signaling pathway, acting on the expression of antioxidant proteins such as HO-1 and SOD1, reducing oxidative stress damage, and playing a protective effect on brain tissue. This study is the first to explore the role of the Nrf2 signaling pathway in the treatment of cerebral infarction by rTMS, which can provide a new theoretical reference for the treatment of clinical cerebral infarction. In the follow-up research, the experiment can be expanded to study more pathways related to cerebral infarction and find methods for targeted therapy.

## Figures and Tables

**Figure 1:** Cerebral ischemia and reperfusion on neuromotor injury in rats. *Note.* (a) Neurological deficit score; (b) removal time of bilateral stickers; (c) balance beam passing time; compared with the sham group, ^*∗*^*p* < 0.05.

**Figure 2:** The expression of Nrf2 and HO-1 and the level of oxidative stress in the brain tissue of experimental cerebral infarction rats. *Note.* (a)-(b) Nrf2 and HO-1 protein expression; (c)-(d) Nrf2 and HO-1 mRNA expression; (e)-(f) oxidative stress level; compared with the sham group, ^*∗*^*p* < 0.05.

**Figure 3:** The effect of repeated transcranial magnetic stimulation on neuromotor function in rats with experimental cerebral infarction. *Note.* (a) Neurological deficit score; (b) removal time of bilateral stickers; (c) balance beam passing time; compared with the sham group, ^*∗*^*p* < 0.05.

**Figure 4:** The effect of repeated transcranial magnetic stimulation on the expression of Nrf2 and HO-1 in the brain tissue of experimental cerebral infarction rats. *Note.* (a)-(b) Nrf2 and HO-1 protein expression; (c)-(d) Nrf2 and HO-1 mRNA expression; compared with the model group, ^*∗*^*p* < 0.05.

**Figure 5:** The effect of repeated transcranial magnetic stimulation on oxidative stress in the brain tissue of experimental cerebral infarction rats. *Note.* (a)-(b) Oxidative stress level; compared with the model group, ^*∗*^*p* < 0.05.

**Table 1:** Related primer sequence.

Primer sequence	Forward (5′—3′)	Reverse (5′—3′)
Nrf2	ATATACGCAGGAGGGAAG	TCCCATCCTCATCACGTAAC
HO-1	TCCCATCCTCATCACGTAAC	CCACGGTCGCCAACAGGAAA
*β*-Actin	CCACGGTCGCCAACAGGAAA	TTTAATGTCACGCACGATTTC

## Data Availability

The datasets used and/or analyzed during the current study are available from the corresponding author upon request.
